The article "A Hybrid Data-Driven Approach for Multistep Ahead Prediction of State of Health and Remaining Useful Life of Lithium-Ion Batteries" was published in 2022. Journal: Comput Intell Neurosci.

# A Hybrid Data-Driven Approach for Multistep Ahead Prediction of State of Health and Remaining Useful Life of Lithium-Ion Batteries

**DOI:** 10.1155/2022/1575303

**Published:** 2022-06-13

**Authors:** Muhammad Umair Ali, Amad Zafar, Haris Masood, Karam Dad Kallu, Muhammad Attique Khan, Usman Tariq, Ye Jin Kim, Byoungchol Chang

**Affiliations:** ^1^Department of Unmanned Vehicle Engineering, Sejong University, Seoul 05006, Republic of Korea; ^2^Department of Electrical Engineering, The Ibadat International University, Islamabad 54590, Pakistan; ^3^Department of Electrical Engineering, University of Wah, Wah Cantt, Pakistan; ^4^School of Mechanical and Manufacturing Engineering (SMME), National University of Science and Technology (NUST), H-12, Islamabad, Pakistan; ^5^Department of Computer Science, HITEC University, Taxila, Pakistan; ^6^College of Computer Engineering and Sciences, Prince Sattam Bin Abdulaziz University, Al-Kharj, Saudi Arabia; ^7^Department of Computer Science, Hanyang University, Seoul 04763, Republic of Korea; ^8^Center for Computational Social Science, Hanyang University, Seoul 04763, Republic of Korea

## Abstract

In this paper, a novel multistep ahead predictor based upon a fusion of kernel recursive least square (KRLS) and Gaussian process regression (GPR) is proposed for the accurate prediction of the state of health (SoH) and remaining useful life (RUL) of lithium-ion batteries. The empirical mode decomposition is utilized to divide the battery capacity into local regeneration (intrinsic mode functions) and global degradation (residual). The KRLS and GPR submodels are employed to track the residual and intrinsic mode functions. For RUL, the KRLS predicted residual signal is utilized. The online available experimental battery aging data are used for the evaluation of the proposed model. The comparison analysis with other methodologies (i.e., GPR, KRLS, empirical mode decomposition with GPR, and empirical mode decomposition with KRLS) reveals the distinctiveness and superiority of the proposed approach. For 1-step ahead prediction, the proposed method tracks the trajectory with the root mean square error (RMSE) of 0.2299, and the increase of only 0.2243 RMSE is noted for 30-step ahead prediction. The RUL prediction using residual signal shows an increase of 3 to 5% in accuracy. This proposed methodology is a prospective approach for an efficient battery health prognostic.

## 1. Introduction

The depletion of fossil fuel resources and issues related to climate change provides a strong impetus to developers to focus on green energy resources, green transportation, and smart grids [1, 2]. Energy storage devices are the core component in the above-mentioned fields. Due to their lightweight, high energy and power density, low self-discharge rate, and long lifecycle, lithium-ion (Li-ion) batteries have superiority among other sources of energy storage devices [3, 4]. However, as the Li-ion battery is one of the system's costly components, it must be handled carefully using an efficient battery management system (BMS) [5]. The role of an intelligent BMS is to manage the battery efficiently and monitor the state of the battery with high accuracy. Li-ion battery malfunctions often lead to functional impairment, degraded performance, or total failure. In recent years, the estimation and prediction of battery state of health (SoH), state of charge (SoC), state of life (SoL), remaining useful life (RUL), and state of function (SoF) gained significant attention for battery health prognostic (BHP) [6–8]. In smart grids, renewable energy systems, and electric vehicles, battery life is one of the most important features to accomplish economic viability. In battery life, battery degradation due to dynamic operational conditions is one of the most critical issues. So early estimation and prediction of battery SoH and RUL are crucial tasks of smart BMS for reliable operation.

The article "A Hybrid Data-Driven Approach for Multistep Ahead Prediction of State of Health and Remaining Useful Life of Lithium-Ion Batteries" was published in 2022. Journal: Comput Intell Neurosci.

Researchers have been working on the Li-ion battery capacity estimation in recent years, as it is the determinative SOH indicator [9, 10]. When the Li-ion battery capacity reaches 80% of its initial capacity, it must be replaced to ensure smooth and reliable operation [11]. However, the battery capacity cannot be measured using any physical sensor, so it is challenging to measure the accurate SoH and RUL. To date, various methodologies have been reported to estimate and predict the SoH and RUL. Based on the literature, these procedures can be categorized as specific model-based methods, data-driven methods, and hybrid approaches [1, 12].

The model-based methods define the battery degradation behavior by using differential, algebraic, or empirical equations. Different researchers presented empirical models [13–15], mechanistic models (also known as chemical models) [16–18], equivalent circuit models [19, 20], and fused models [21] to capture the battery degradation behavior. Hu et al. [22] presented a model-based method for coestimation of SoC and SoH of Li-ion batteries. The utilized fractional-order battery model is identified using a hybrid optimization algorithm, and the model shows a steady-state error of less than 1%. In their subsequent work [23], the authors utilized incremental capacity analysis to determine the SoH of the electric taxi. Their proposed methodology has the root mean square error of 0.0204. Although the model-based methods have good accuracy, they still have some drawbacks. The empirical and equivalent circuit techniques are easy to build a model. Still, it only accurately measures the short-term states due to changing parameters during the cycling process. However, filtering algorithms are utilized to update the model parameters at the cost of the high complexity of the system. Similarly, mechanistic models also have increased complexity and require expert knowledge to build the model [1]. It is also difficult to build these models in noisy/uncertain environments.

The article "A Hybrid Data-Driven Approach for Multistep Ahead Prediction of State of Health and Remaining Useful Life of Lithium-Ion Batteries" was published in 2022. Journal: Comput Intell Neurosci.

The data-driven methods require only Li-ion battery sensor data (voltage, current, and temperature) to predict the SoH and RUL [24]. Different machine learning algorithms were used to build the connection between operation data and battery degradation. Compared to model-based approaches, it does not require any complex physical model; it only builds a weight vector based upon its training data. Tian et al. [25] proposed a deep learning sequence to sequence model to predict the capacity degradation of the Li-ion battery. The authors used the data of one cycle of the Li-ion battery for multistep (100, 200, and 300 cycles) ahead prediction. In another study [26], for the prediction of the entire charging curve, a deep neural network was trained with discrete sections of the charging curves as input. Thirty data points were collected as input in less than 10 minutes to train the deep learning model. Wang et al. [27] proposed a data-driven approach to diagnosing the abnormality in the battery charging capacity. These techniques need historical data to train the model. In the past, relevance vector machine, logic regression, and support vector machine have been reported to predict the RUL [28]. In a study [29], the authors presented the Bayesian model to predict the RUL of Li-ion batteries under dynamic operating conditions. They showed that their proposed model had better prediction accuracy as compared to the support vector machine. Tang et al. [30] proposed a balancing current ratio-based SOH predictor for series-connected cells in a battery pack. Liu et al. [31] proposed a two-stage trajectory model to determine the future aging trajectory with uncertainty quantification. Wang et al. [32] proposed another variant of the Bayesian model to predict the RUL. Neural network [33, 34], autoregressive fused model [35], and Box-Cox transformation [36] were also utilized to estimate the battery capacity. In all aforementioned literature, they directly neglect the effect of fluctuation and local regeneration phenomena in the capacity, affecting prediction accuracy. A Gaussian process functional regression model was proposed to tackle the issue of local capacity regeneration [37]. A variant of recurrent neural network (long short-term memory) was proposed to predict the Li-ion battery capacity [38]. Their experimental results show an average error of 0.0765 Ah (2.46%). In a recent study [39], a hybrid method based upon long short-term memory and Gaussian process regression (GPR) has been proposed to predict the capacity and RUL of Li-ion batteries. The GPR and long short-term memory were utilized to capture local regeneration and global capacity degradation trend. They also predict the battery RUL for multistep ahead. The maximum noted error was less than 1.8%. However, it has been observed that the battery local fluctuation and regeneration have a significant impact on the multistep ahead prediction of SoH and RUL. Therefore, further research is needed to predict q-step ahead SoH and RUL with high accuracy.

The article "A Hybrid Data-Driven Approach for Multistep Ahead Prediction of State of Health and Remaining Useful Life of Lithium-Ion Batteries" was published in 2022. Journal: Comput Intell Neurosci.

Driving by the desire to increase the BMS reliability and improve battery safety. In this study, a novel hybrid method consisting of multiscale kernel recursive least square (KRLS) and GPR is proposed for the q-step ahead SoH prediction of Li-ion battery. To be more explicit, the following are the proposed approach's key contributions:

- The empirical mode decomposition (EMD) method is employed to split the local generation, global battery degradation, and other fluctuations.
- The KRLS with an autoregressive moving average with exogenous signals (ARMAX) model is recursively used to predict global battery degradation. GPR is applied to track the local fluctuation and regeneration of the Li-ion battery.
- Finally, the prediction of KRLS and GPR ensemble to obtain the final predicted SoH.
- The RUL is predicted using SOH, intrinsic mode functions (IMFs), and a residual value of the battery data.
- The suggested approach is validated using various online datasets (NASA and CALCE).
- Experimental results and comparative analysis reveal the effectiveness and supremacy of the proposed methodology, respectively.

## 2. State of Health of Lithium-Ion Battery

Li-ion battery is a highly nonlinear and complex electrochemical system, which significantly impacts its health under dynamic operating conditions. SoC, SoH, SoL, and RUL are the different parameters primarily used to predict the health of Li-ion batteries [40, 41]. SoH is one of the essential components of the BHP system [42]. The most widely accepted definition of SoH of the Li-ion battery can be stated as the ratio of battery capacities at the *kth* cycle and initial cycle. In other words, it can be explained using the following mathematical equation:

(1) $$\begin{array}{c} SoH_{k}=\frac{Q_{k}}{Q_{o}}\times 100\%, \end{array}$$

where *SoH*_*k*_ is the SoH at *kth* cycle, and *Q*_*k*_ and *Q*_*o*_ are the battery capacities at *kth* cycle and initial cycle, respectively. However, battery degradation can occur in the cathode and anode. Therefore, a scalar SOH is not sufficient. For further details, see [43, 44].

The article "A Hybrid Data-Driven Approach for Multistep Ahead Prediction of State of Health and Remaining Useful Life of Lithium-Ion Batteries" was published in 2022. Journal: Comput Intell Neurosci.

## 3. Methodology

In this section, the framework of the proposed methodology has been explained in detail.

### 3.1. Empirical Mode Decomposition (EMD)

The EMD is a very efficient tool for analyzing highly dynamic signals; it decomposes the nonstationary and nonlinear signals into different oscillatory components known as series of IMFs and residuals. Owing to its extraordinary abilities, it has been implemented in other fields (e.g., image processing, vibration, rotating machinery). Huang et al. [45] discussed the EMD approach in more detail. In the EMD approach, the IMFs should satisfy the following condition after decomposition.

1. The mean value of upper and lower envelopes must be equal to 0 at any instant.
2. In the whole time series input dataset, the no. of zero crossings and the no. of extrema must be equal to 1 or 0.

In this work, it is considered that the local fluctuation and regeneration phenomena in original SoH signals are the high-frequency components, and global SoH degradation is the low-frequency SoH signal. This signal decomposition is also known as the sifting phenomenon. After finding all the extreme values (minima and maxima) in the input signal (*x*_*k*_), then connect all the local minimum and maximum values using a spline line to develop a lower (*e*_*k*,lower_) and upper (*e*_*k*,upper_) envelope, respectively. After this, compute the local mean of both envelopes by using the following equation:

(2) $$\begin{array}{c} m_{k}=\frac{e_{k,\text{upper}}+e_{k,\text{lower}}}{2}. \end{array}$$

Determine the difference (*D*) between the *x*_*k*_ and the mean value (*m*_*k*_).

(3) $$\begin{array}{c} D=x_{k}-m_{k}. \end{array}$$

After calculating the difference, check whether *D* fulfills the IMFs condition, as discussed above. If it meets all the conditions to be an IMF signal, remove it from the *x*_*k*_ to obtain the residual signal (res).

(4) $$\begin{array}{c} res_{k,1}=x_{k}-D. \end{array}$$

Repeat all the steps until the residue meets the stopping criteria. All the information on local fluctuation and regeneration has been saved in IMFs, and monotonous residue contains the information on the global degradation of SoH [46]. By adding all the IMFs and monotonous residue, the original input signal can be described as follows:

(5) $$\begin{array}{c} x_{k}=\sum_{j=1}^{n}IMF_{k,n}+res_{k,n}. \end{array}$$

In this work, the wavelet and signal processing toolbox of MATLAB® was utilized to perform the EMD. The flowchart of the working of EMD is shown in Figure 1.

The article "A Hybrid Data-Driven Approach for Multistep Ahead Prediction of State of Health and Remaining Useful Life of Lithium-Ion Batteries" was published in 2022. Journal: Comput Intell Neurosci.

### 3.2. Kernel Recursive Least Square

In this work, the ARMAX model is used to predict the SoH of the battery. The ARMAX model can be represented using the following equation [47]:

(6) $$\begin{array}{c} y_{k}=\sum_{m=1}^{M}\alpha_{m}y_{\left(k-m\right)}+\sum_{n=1}^{N}\beta_{n}u_{\left(k-n\right)}+\gamma .1+\varepsilon_{k}, \end{array}$$

where *y* and *u* are the measured signal and desired response, respectively. *α*, *β*, and *γ* are the model coefficients, which have to be estimated recursively. *ε* represents the zero-mean Gaussian noise. *M* and *N* are the order of the system and the input. The above mathematical model can be written in a simplified form as follows:

(7) $$\begin{array}{c} y_{k}=\varphi_{k}^{T}\theta_{k}+e_{k}, \end{array}$$

(8) $$\begin{array}{c} \varphi_{k}^{T}=\left[y_{k-1}\cdots y_{k-M}u_{k-1}\cdots u_{k-N}1\right], \end{array}$$

(9) $$\begin{array}{c} \theta_{k}=\left[\alpha_{1}\cdots \alpha_{M}\beta_{1}\cdots \beta_{N}\gamma \right], \end{array}$$

where *φ*^*T*^ is the transpose of the regression vector. The KRLS method can be utilized to determine the unknown coefficients of the above equation. The cost function can be expressed by the following equations:

(10) $$\begin{array}{c} \underset{\theta_{k}}{\min}J_{KRLS}=\sum_{k=1}^{n}\lambda_{n-k}{\left|y_{k}-\kappa {\left(\varphi_{k},.\right)}^{T}\theta_{k-1}\right|}^{2}+R\lambda^{N}{\left\|\theta_{k-1}\right\|}_{H}^{2}, \end{array}$$

(11) $$\begin{array}{c} \phi_{k}={\left[\kappa \left(\varphi_{1},.\right)\kappa \left(\varphi_{2},.\right)\cdots \kappa \left(\varphi_{k},.\right)\right]}^{T}, \end{array}$$

where Mercer kernel is represented by *κ*. *ϕ*, *R*, *H*, and *λ* are the kernel matrix, regularization factor (always taken as a positive number), reproducing kernel Hilbert space (RKHS), and the forgetting factor, respectively. The most commonly used kernel for prediction are the Gaussian kernel *κ*(*φ*, *φ*^″^)=exp(−‖*φ* − *φ*^″^‖/2*σ*^2^), polynomial kernel *κ*(*φ*, *φ*^″^)=(*φ*^*T*^*φ*^″^+*c*)^*p*^, and sigmoid kernel *κ*(*φ*, *φ*^″^)=tanh(*s*(*φ*^*T*^*φ*^″^)+*t*) [48], where *σ*, *φ*^″^, *c*, and *p* are the scaling factor, latest upcoming data, positive valued constant, and polynomial order, respectively. *s* and *t* both are positive constants. In this work, all the kernel function was implemented. The presented results are of the polynomial kernel, which shows the best accuracy.

The KRLS method works by mapping input data into high dimension RKHS. In this process, the linear inner product changes into RKHS by simply replacing the inner product with kernels [49, 50]. The linear algorithms can then be used to solve the transformed feature space (RKHS). The unique global solution is the salient feature of kernel-based methods [51]. Additionally, if the input data is highly nonlinear, the linear regression techniques fail to model it accurately. Kernel-based algorithms can easily tackle this issue by mapping the nonlinear data into high dimension linear feature space. Because of the high dimensionality of data in RKHS, it experiences overfitting problems. This issue can be resolved by penalizing it to the L2 norm, as shown in (10) [52], which can be solved and updated as follows [53]:

(12) $$\begin{array}{c} \theta_{k}=\phi_{k}{\left[R\lambda +\phi_{k}^{T}\phi_{k}\right]}^{-1}y_{k},\theta_{k}=\phi_{k}a_{k},a_{k}=Q_{k}y_{k},\\ Q_{1}={\left[R\lambda +\kappa \left(\varphi_{1},\varphi_{1}\right)\right]}^{-1},a_{1}=Q_{1}y_{1},\\ K_{k}=K_{k-1}^{T}\kappa \left(\varphi_{1},.\right)={\left[\kappa \left(\varphi_{1},\varphi_{k}\right)\kappa \left(\varphi_{2},\varphi_{k}\right)\cdots \kappa \left(\varphi_{k-1},\varphi_{k}\right)\right]}^{T},\\ z_{k}=Q_{k-1}K_{k},\\ \delta_{k}=R\lambda +\kappa \left(\varphi_{k},\varphi_{k}\right)-z_{k}^{T}K_{k},\\ Q_{k}=\delta_{k}^{-1}\left[\begin{array}{cc} Q_{k-1}\delta_{k}+z_{k}z_{k}^{T} & -z_{k}\\ -z_{k} & 1 \end{array}\right],\\ e_{k}=y_{k}-K_{k}^{T}a_{k-1},\\ a_{k}=\left[\begin{array}{c} a_{k-1}-z_{k}\delta_{k}^{-1}e_{k}\\ \delta_{k}^{-1}e_{k} \end{array}\right]. \end{array}$$

The approximate linear dependency criteria are used to reduce the computation complexity of KRLS due to an increase in observations [54]. In this work, the KRLS coupled with approximate linear dependency has been employed using MATLAB®. To estimate the model capacity $\left({\hat{y}}_{k}\right)$, (7) can be written as follows:

(13) $$\begin{array}{c} {\hat{y}}_{k}=\varphi_{k}^{T}{\hat{\theta }}_{k}+e_{k}. \end{array}$$

(13) can be modified for q-step ahead prediction $\left({\hat{y}}_{k+q}\right)$ as follows:

(14) $$\begin{array}{c} {\hat{y}}_{k+q}=\varphi_{k+q}^{T}{\hat{\theta }}_{k}+e_{k}. \end{array}$$

The article "A Hybrid Data-Driven Approach for Multistep Ahead Prediction of State of Health and Remaining Useful Life of Lithium-Ion Batteries" was published in 2022. Journal: Comput Intell Neurosci.

### 3.3. Gaussian Process Regression

A GPR is an effective approach to solving nonlinear regression and classification problems [55, 56]. GPR is a probabilistic nonparametric model, which combines different variables; these combinations are defined by the probability distribution (*f*(*x*)). The GPR model can be described by its mean and covariance (kernel) function as follows:

(15) $$\begin{array}{c} f\left(x\right)∼GPR\left(m\left(x\right),k\left(x,x^{\prime }\right)\right), \end{array}$$

where *m*(*x*) and *k*(*x*, *x*′) are the mean and covariance functions, respectively. The *m*(*x*) function is mainly assumed as zero. The relation between input and output can be expressed as follows:

(16) $$\begin{array}{c} y=f\left(x\right)+\varepsilon , \end{array}$$

where *ε* is the additive noise, which has zero mean and variance of *σ*_*n*_^2^.

(17) $$\begin{array}{c} \varepsilon ∼N\left(0,\sigma_{n}^{2}\right). \end{array}$$

By using (16), the likelihood can be written as follows:

(18) $$\begin{array}{c} p\left(y|f\right)=N\left(y|f,\sigma_{n}^{2}I\right)y, \end{array}$$

where *y*=[*y*_1_, *y*_2_, *y*_3_ … *y*_*n*_]^*T*^, *f*=[*f*(*x*_1_), *f*(*x*_2_), *f*(*x*_3_) … *f*(*x*_*n*_)], and *I* is the *M* × *M* unit matrix. According to [57], the marginal distribution of *p*(*f*) can be written as follows:

(19) $$\begin{array}{c} p\left(f\right)=N\left(f\;|\;0,K\right), \end{array}$$

where *K*=*k*(*x*_*i*_, *x*_*j*_), using (18) and (19).

(20) $$\begin{array}{c} p\left(y\right)=\int p\left(y|f\right)p\left(f\right)\text{d}f=N\left(f|0,K_{y}\right), \end{array}$$

where *K*_*y*_=*K*+*σ*_*n*_^2^*I*, for the prediction of the target value (*y*_*∗*_) for the updated input value, the joint distribution over *y*_1_, *y*_2_, *y*_3_,…*y*_*m*_, *y*_*∗*_ can be written as follows:

(21) $$\begin{array}{c} \left[\begin{array}{c} y\\ y_{*} \end{array}\right]=\left(\left[\begin{array}{c} f\\ f_{*} \end{array}\right]+\left[\begin{array}{c} \varepsilon \\ \varepsilon_{*} \end{array}\right]\right):N\left(0,\left[\begin{array}{c} \begin{array}{c} K_{y}\\ k_{*}^{T} \end{array}\\ \begin{array}{c} k_{*}\\ k_{{*}^{*}}+\sigma_{n}^{2} \end{array} \end{array}\right]\right), \end{array}$$

where *f*_*∗*_=*f*(*x*_*∗*_) is the latent function corresponding to its input *x*_*∗*_ and noise *ε*_*∗*_. *k*_*∗*_=[*k*(*x*_*∗*_, *x*_1_), *k*(*x*_*∗*_, *x*_2_), *k*(*x*_*∗*_, *x*_3_),…,*k*(*x*_*∗*_, *x*_*M*_)]^*T*^ and *k*_*∗∗*_=*k*(*x*_*∗*_, *x*_*∗*_). The predictive distribution *p*(*y*_*∗*_|*y*) is the Gaussian distribution, which has the following characteristics:

(22) $$\begin{array}{c} m\left(x_{*}\right)=k_{*}^{T}K_{y}^{-1}y,\\ \sigma \left(x_{*}\right)=k_{**}-k_{*}^{T}K_{y}^{-1}k_{*}+\sigma_{n}^{2}. \end{array}$$

The *K*_*y*_^−1^ can be calculated using Cholesky decomposition [58]. The covariance (kernel) function is a very critical component in the prediction process. The rational quadratic kernel functions are used for the prediction [39].

### 3.4. Proposed Methodology

In this work, EMD, KRLS, and GPR-based fused battery SoH prediction models have been proposed. The framework of the proposed approach is shown in Figure 2.

The raw battery sensor data is passed through the Savitzky-Golay filter to reduce the measurement noise error [59]. The filter is implemented using the MATLAB® tool *sgolayfilt*. After that, the battery SoH was calculated using (1). The EMD technique is utilized to decompose the battery SoH in IMFs and its residual signals, as discussed in Section 3.1. The KRLS and GPR methodology was adopted to track the global degradation and local regeneration phenomenon in the Li-ion battery, respectively. Finally, the predicted IMFs and residuals were ensembled to get the predicted SoH. When the predicted SoH exceeds the battery end of life (EOL), the RUL will be predicted. Percentage fitting (FIT) and root mean square error (RMSE) were utilized to evaluate the performances of SoH prediction.

(23) $$\begin{array}{c} \text{FIT}=100\left(1-\sqrt{\frac{\sum_{k=1}^{N}{\left(y_{k}-{\hat{y}}_{k}\right)}^{2}}{\sum_{k=1}^{N}{\left(y_{k}-\text{mean}\left(y_{k}\right)\right)}^{2}}}\right),\\ \text{RMSE}=\sqrt{\frac{1}{N}\sum_{k=1}^{N}{\left(y_{k}-{\hat{y}}_{k}\right)}^{2}}. \end{array}$$

where *y*_*k*_ and ${\hat{y}}_{k}$ are the original and estimated output, and *N* is the total number of samples.

The article "A Hybrid Data-Driven Approach for Multistep Ahead Prediction of State of Health and Remaining Useful Life of Lithium-Ion Batteries" was published in 2022. Journal: Comput Intell Neurosci.

In this study, to examine the accuracy of RUL prediction, the following testing standard has been followed:

(24) $$\begin{array}{c} \text{Accuracy}\left(\text{\%}\right)=\left(1-\frac{\left|RUL_{\text{actual}}-RUL_{\text{predicted}}\right|}{RUL_{\text{actual}}}\right)\times 100. \end{array}$$

## 4. Experimental Data and Results

In this section, the proposed methodology's distinctiveness is evaluated using NASA's online available data source [60]. The details of different battery datasets are presented in Table 1. All the processing is done on MATLAB 2021 ® with the personal computer having the specification of Intel(R) Core (TM) i7-10700 CPU @ 2.90 GHz processor with 32 GB RAM, 1 TB SSD, and a 64-bit Windows 10 Pro operating system (OS).

The cyclic aging experiments were carried out on all NASA batteries using a programmed electric load, adjustable temperature chamber, and electric supply [61]. The discharge current and temperature of all the Li-ion batteries are shown in Table 1. Further details of the experimental setup can be found in [61]. The SoH trends of all Li-ion batteries can be seen in Figure 3.

After collecting battery data through transducers, it passes through the Savitzky-Golay filter. The filter reduced the measurement noise error. The EMD technique decomposes the Li-ion battery SoH into residual and IMFs signals, as shown in Figure 4.

The prediction results of Li-ion batteries B0005. B0006, B0018, B0055, and B0056 using the proposed technique (EMD, KRLS, and GPR) are shown in Figure 5, respectively.

For the comparison between the proposed and other methodologies such as solo GPR, solo RLS, EMD + GPR, and EMD + KRLS, the results are presented in Figure 6.

The article "A Hybrid Data-Driven Approach for Multistep Ahead Prediction of State of Health and Remaining Useful Life of Lithium-Ion Batteries" was published in 2022. Journal: Comput Intell Neurosci.

To further validate the model, another available online dataset of the Center for Advanced Life Cycle Engineering (CALCE) at the University of Maryland is used for prediction [62]. The Arbin BT2000 system with a temperature-controlled chamber was used to perform all cycling tests on the CALCE battery dataset (CX2-16). The CX2-16 battery was drained at 1.1 A steady current, for further information on the experimental setting, see [39, 61]. 60% of the data is used for the training and the rest for the Li-ion battery capacity prediction (CX2-16). The prediction results are shown in Figure 7.

The FIT of 1-step ahead prediction of the proposed methodology for all datasets is shown in Figure 8.

The q-step ahead prediction of the proposed methodology is shown in Figure 9 (for B0018), and the RMSE results of all datasets are presented in Table 2, respectively.

The q-step ahead prediction comparison of proposed and other methodologies is illustrated in Figure 10.

The results of RUL prediction accuracy against different parameters have been presented in Tables 3–7 for the Li-ion batteries. For all Li-ion battery datasets, the RUL is predicted at various cycle numbers to check the accuracy. The comparison of the proposed approach with another state-of-the-art study is shown in Table 8.

## 5. Discussion

In this work, a BHP model is proposed to avoid unexpected battery failures. As discussed earlier, the accurate and early SoH prediction of Li-ion batteries is one of the main components of intelligent BMS.

The basic framework of the proposed approach is shown in Figure 2. After the filtration step, the EMD technique divides the SoH of the Li-ion battery into its global degradation (residual) and local regeneration (IMFs) (see Figure 4). The EMD technique consumes 0.54 ms and 2.31 ms to decompose the data of Li-ion batteries B0055 (102 data points) and CX2-16 (1998 data points), respectively. The residual shows the actual SoH degradation of the Li-ion battery (Figure 4). Meanwhile, all local regeneration points of the original SoH were captured by all IMFs. The one-step-ahead prediction results of Li-ion batteries B0005. B0006, B0018, B0055, and B0056 are shown in Figure 5. 110 battery cycles out of 168 were used to train the model for B0005 and B0006, as shown in Figures 5(a) and 5(b). The KRLS effectively tracks the residual values without any significant error, as shown in Figure 5. The GPR was utilized to predict the IMFs signal of the batteries, and it shows good tracking ability, also reported in [39]. The proposed methodology shows similar accuracy in the case of B0018. 80 out of 127 samples were used to train the models (see Figure 5(c)). In [61], the author used B0005, B0006, and B0018 to validate his proposed multiscale logic regression (LR) and GPR model. The results showed the maximum RMSE of 0.8 for 1-step ahead prediction; in comparison, our proposed methodology shows the maximum RMSE of 0.284 for the mentioned dataset. The data of Li-ion batteries B0055 and B0056 was noisy because these batteries were operated at 4°C. The proposed methodology still shows high accuracy in the presence of perturbation, as seen in Figures 5(d) and 5(e). Figure 6 reported the comparison results; the solo GPR has poor tracking capability and shows a significant prediction error. In contrast, EMD with KRLS has shown the second-best prediction accuracy after the proposed approach. For the CALCE dataset, 1200 data points from 1998 were used to train the model. The prediction RMSE was just 0.64 for the whole prediction of 798 data points (see Figure 7). The proposed method predicts 1-step ahead values with high accuracy (Figure 8). The SoH fitting accuracy of B0055 and B0056 is on a bit lower side due to high perturbation in the measured signal. However, it still shows better accuracy as compared to [61].

The article "A Hybrid Data-Driven Approach for Multistep Ahead Prediction of State of Health and Remaining Useful Life of Lithium-Ion Batteries" was published in 2022. Journal: Comput Intell Neurosci.

For all the datasets, for q-step ahead prediction, 5, 10, 15, 20, 25, and 30 steps ahead prediction was carried out. The graphical presentation of the q-step ahead of the Li-ion battery (B0018) is shown in Figure 9. It can be observed that the proposed methodology shows high accuracy even in the case of a 30-step ahead prediction (see Table 2). The RMSE of the 1-step prediction of B0006 was 0.2299, while it shows only a small increase of 0.2243 in RMSE for the 30-step ahead prediction. In some cases, the prediction RMSE reduces with the increase of the value of the ahead prediction step. In the case of B0005, the 0.2823 RMSE was noted at 5-step ahead prediction, while the RMSE at 10-step ahead prediction is just 0.2296, which is 0.0527 lesser than the 5-step ahead prediction error. At 5-step ahead prediction of Li-ion battery (B0005), there was a regeneration point to predict, which is why the RMSE was more at 5-step than 10-step. The maximum RMSE of 1.1021 was noted for Li-ion battery (B0055) at 30-step ahead prediction under a perturbated environment. The q-step ahead prediction comparison analysis reveals the effectiveness and distinctiveness of the proposed methodology under q-step ahead prediction (see Figure 10).

For a smart BMS, the early accurate prediction of Li-ion battery RUL is one of the key components for safe and reliable operation. Different features were used to predict the RUL at different cycle numbers using the proposed robust model in this work. Predicted SoH, IMFs, and residual were used to estimate the future RUL of the Li-ion battery. All the RUL prediction results of Li-ion batteries are tabulated in Tables 3–7. For B0005 and B0006, the RUL prediction was started at cycles 50 to 120 with a difference of 5 cycles; it can be observed in Table 3 that the RUL accuracy was just 75.59% at the 50^th^ cycle using SoH as the predictor, while residual has the accuracy of 99.21% at the same point. In [61], the RUL prediction accuracy of just 79.84% was observed at the 50^th^ cycle. The RUL prediction accuracy increased with the prediction point (i.e., at 110 cycles, the RUL prediction accuracy was 94.57%). Similarly, a prediction error of 3.3% was noted in [39]. The residual has the minimum RUL prediction accuracy of 96.06% at the 90^th^ cycle. In comparison, SoH has an accuracy of 96.85% at the same point. The accuracy of IMFs was far below the accuracy of SoH and residual, which is also reflected in the results. The average RUL prediction accuracy using residual and SoH as a feature was 97.53% and 94.12%, respectively. It can be concluded that the prediction of RUL using residual value has better accuracy as compared to other parameters. Similar results can be observed for all other batteries (see Tables 4–7). For Li-ion battery CX2-16, the average RUL prediction accuracy was 99.51%. An average absolute error of only 3, 12, and 3 cycles is noted for the Li-ion battery B0005, B0006, and B0018, which is 13, 10, and 2 cycles lesser than the other study [61] (see Table 8). Hence, after extensive experimentation and comprehensive analysis, it can be concluded that the proposed trained model predicts the SoH and RUL with high accuracy.

The article "A Hybrid Data-Driven Approach for Multistep Ahead Prediction of State of Health and Remaining Useful Life of Lithium-Ion Batteries" was published in 2022. Journal: Comput Intell Neurosci.

## 6. Limitations and Future Perspectives

The presented technique for predicting battery health might be employed to develop a BMS. The prediction model, on the other hand, is validated in a controlled environment, such as constant charging/discharging current and temperature. In contrast, the operation circumstances fluctuate substantially throughout cycles, causing the battery to deuterate in numerous phases. Therefore, the performance of the proposed approach must be checked under dynamic conditions. Furthermore, the RUL prediction of a single battery cell is solely considered in this study. However, in a battery pack, numerous cells are connected in series/parallel. Because of the unequal aging of the battery cells caused by the temperature differential, the battery pack RUL prediction must be investigated with uncertainty quantification in the future.

## 7. Conclusion

In this work, the battery health predictor has been proposed to reduce the chances of unexpected battery failures. To address the issue of accurate prediction for local regeneration in the SoH signal, the EMD technique was employed to decompose data into low and high-frequency signals. The recursive KRLS method was utilized to track the global battery degradation and GPR to predict the local fluctuation and regenerations points with high accuracy. The proposed methodology shows above 91% fitting accuracy at 1-step ahead prediction under a normal environment. It has the maximum RMSE of 1.1021 at 30-step ahead prediction under a perturbated environment. The comparison analysis also illustrated that the proposed methods are more effective and accurate. Furthermore, the results show that the RUL prediction using the residual has 3 to 5% higher accuracy than the RUL prediction using SoH. It means that the proposed technique can be utilized to design the battery health prognostics.

The article "A Hybrid Data-Driven Approach for Multistep Ahead Prediction of State of Health and Remaining Useful Life of Lithium-Ion Batteries" was published in 2022. Journal: Comput Intell Neurosci.

## Figures and Tables

**Figure 1:** Flowchart of EMD.

**Figure 2:** A framework of the proposed methodology.

**Figure 3:** SoH degradation of different batteries.

**Figure 4:** Decomposition of Li-ion battery (B0018).

**Figure 5:** Prediction results of Li-ion battery using proposed approach: (a) B0005; (b) B0006; (c) B0018; (d) B0055; (e) B0056.

**Figure 6:** 1-step ahead prediction comparison of different techniques.

**Figure 7:** The prediction results of Li-ion battery (CX2-16).

**Figure 8:** Percentage fitting of the proposed methodology for 1-step ahead prediction.

**Figure 9:** Q-step ahead prediction of Li-ion battery (B0018).

**Figure 10:** q-step ahead prediction comparison (B0018).

**Table 1:** Details of the dataset used for prediction.

Battery type	Battery no.	Lower cutoff voltage (V)	Upper cutoff voltage (V)	Charging current (A)	Discharging current (A)	Operating temperature (°C)	New battery capacity (ah)	Total no. of cycle	End of life
Li-ion 18650	B0005	2.7	4.2	1.5	2	24	1.86	168	127
	B0006	2.5				24	2.04	168	127
	B0018	2.5				24	1.85	127	97
	B0055	2.5				4	1.32	102	70
	B0056	2.7				4	1.34	102	70

**Table 2:** RMSE of proposed technique at q-step ahead prediction.

	1_step	5_step	10_step	15_step	20_step	25_step	30_step
B0005	0.2723	0.2823	0.2296	0.2877	0.3016	0.334	0.4125
B0006	0.2299	0.2341	0.3283	0.3651	0.4023	0.4183	0.4542
B0018	0.284	0.3135	0.3455	0.3582	0.3452	0.4243	0.4997
CX2_16	0.6444	0.6654	0.6723	0.6776	0.7293	0.7322	0.7837
B0056	0.8129	0.8239	0.8546	0.8927	0.9321	0.9567	0.9912
B0055	0.9025	0.9491	0.9412	0.9715	1.0012	1.0123	1.1021

**Table 3:** RUL prediction accuracy (%) for B0005.

RUL Parameters	Cycle numbers														
	50	55	60	65	70	75	80	85	90	95	100	105	110	115	120
SOH	75.59	84.25	88.19	92.13	94.49	96.85	98.43	100	96.85	96.85	99.21	96.06	99.21	96.85	96.85
IMF 1	85.83	37.8	59.84	72.44	72.44	64.57	72.44	73.23	86.61	75.59	95.28	82.68	69.29	96.06	97.64
IMF 2	62.2	85.83	62.2	66.93	74.02	75.59	88.19	59.06	93.7	86.61	65.35	87.4	92.91	87.4	70.08
IMF 3	69.29	71.65	74.8	77.95	80.31	81.89	91.34	88.98	87.4	85.83	88.98	95.28	100	98.43	100
Residual	99.21	99.21	98.43	97.64	97.64	96.85	96.85	96.85	96.06	96.06	96.85	96.85	97.64	97.64	99.21

The article "A Hybrid Data-Driven Approach for Multistep Ahead Prediction of State of Health and Remaining Useful Life of Lithium-Ion Batteries" was published in 2022. Journal: Comput Intell Neurosci.

**Table 4:** RUL prediction accuracy (%) for B0006.

RUL Parameters	Cycle numbers														
	50	55	60	65	70	75	80	85	90	95	100	105	110	115	120
SOH	97.64	98.43	89.76	84.25	81.1	81.89	85.83	84.25	84.25	94.49	92.13	97.64	93.7	95.28	96.06
IMF 1	100	48.82	70.87	75.59	81.89	81.1	86.61	93.7	73.23	66.14	74.02	79.53	90.55	80.31	94.49
IMF 2	93.7	99.21	40.16	46.46	48.82	68.5	94.49	11.81	98.43	33.07	98.43	14.17	22.05	18.9	32.28
IMF 3	10.24	20.47	8.66	18.9	40.16	37.8	14.96	30.71	72.44	77.17	59.84	52.76	65.35	85.04	99.21
Residual	96.06	93.7	91.34	89.76	88.98	88.19	87.4	88.19	88.98	89.76	91.34	92.91	94.49	96.85	98.43

**Table 5:** RUL prediction accuracy (%) for B0018.

RUL Parameters	Cycle numbers											
	40	45	50	55	60	65	70	75	80	85	90	95
SOH	97.94	94.85	80.41	92.78	92.78	97.94	93.81	98.97	96.91	95.88	98.97	96.91
IMF 1	78.35	13.4	78.35	30.93	80.41	78.35	70.10	97.94	96.91	91.75	84.54	85.57
IMF 2	04.12	78.35	41.24	53.61	84.54	80.41	78.35	95.88	91.75	90.72	49.48	75.26
Residual	96.91	100	98.97	98.97	100	97.94	95.88	94.85	93.81	93.81	95.88	98.97

**Table 6:** RUL prediction accuracy (%) for B0055.

RUL Parameters	Cycle numbers							
	30	35	40	45	50	55	60	65
SOH	62.86	58.57	62.86	82.86	97.14	84.29	88.57	91.43
IMF 1	44.29	02.86	21.43	68.57	45.71	38.57	60.00	68.57
IMF 2	30.00	14.29	18.57	30.00	75.71	22.86	57.14	64.29
IMF 3	74.29	02.86	44.29	25.71	82.86	75.71	27.14	21.43
IMF 4	05.71	34.29	72.86	98.57	82.86	80.00	85.71	92.86
Residual	84.29	84.29	84.29	84.29	85.71	88.57	91.43	95.71

**Table 7:** RUL prediction accuracy (%) for CX2-16.

RUL Parameters	Cycle numbers													
	1330	1360	1390	1420	1450	1480	1510	1540	1570	1600	1630	1660	1690	1720
SOH	92.39	97.61	95.74	95.4	93.98	90.17	77.27	91.76	89.89	99.83	81.88	82.95	81.14	84.32
IMF 1	90.51	86.7	81.42	58.64	81.53	79.32	51.76	86.14	74.09	86.65	31.99	67.16	44.72	70.74
IMF 2	87.61	96.14	95.17	95.17	99.66	91.93	71.48	97.22	74.66	88.07	89.89	89.03	91.31	80.34
IMF 3	91.7	69.03	49.66	59.03	97.95	81.42	95.8	72.5	80.68	21.65	72.9	52.33	43.47	72.78
IMF 4	65.85	43.64	1.31	74.82	10.97	15.63	67.84	30.45	73.41	57.73	37.9	16.7	22.95	36.7
IMF 5	31.31	42.73	95.4	31.7	17.9	55.63	84.55	47.33	45.34	72.1	94.66	72.9	64.94	70.34
IMF 6	53.18	72.44	64.94	14.32	35.8	82.22	77.33	45.17	23.47	12.73	11.82	19.43	34.43	55.4
Residual	98.52	98.86	99.2	99.49	99.72	99.94	99.89	99.72	99.6	99.55	99.55	99.6	99.72	99.89

The article "A Hybrid Data-Driven Approach for Multistep Ahead Prediction of State of Health and Remaining Useful Life of Lithium-Ion Batteries" was published in 2022. Journal: Comput Intell Neurosci.

**Table 8:** Comparison of the RUL prediction of the proposed approach with another study.

Prediction starting point	Proposed			Yu [61]		
	B0005	B0006	B0018	B0005	B0006	B0018
50	1	5	1	26	39	18
60	2	11	0	24	40	8
70	3	14	4	18	23	7
80	4	16	6	14	16	5
90	5	14	4	13	14	4
100	4	11	—	10	1	-
110	3	—	—	7	—	—
Average absolute error	**3**	**12**	**3**	16	22	5

## Data Availability

The data used in this work are collected from the following public websites: https://ti.arc.nasa.gov/tech/dash/groups/pcoe/prognostic-data-repository/ and https://web.calce.umd.edu/batteries/data.htm.
